This article has been retracted.

# Clinical Nursing Experience Sharing of Patients with Severe Lung Injury Caused by Gas Poisoning

**DOI:** 10.1155/2022/4888524

**Published:** 2022-04-04

**Authors:** Lixia Li

**Affiliations:** Department of Nursing, Wulanchabu Medical College, Wulanchabu, Inner Mongolia 012000, China

## Abstract

**Objective:**

To study the first aid and nursing methods of patients with coal gas poisoning and explore the nursing effect.

**Method:**

The clinical data of 50 patients with carbon monoxide poisoning admitted to the emergency department of our hospital from February 2011 to August 2016 were retrospectively analyzed. The patients with severe toxic pulmonary edema were selected as the sample population, and all patients were equally divided by drawing lots. The two groups were divided into the study group and control group. The patients in the control group were given routine nursing intervention, while the patients in the study group were given routine nursing intervention. After the timely treatment of doctors in our hospital and the careful nursing of nursing staff, 45 patients in 50 patients were cured and discharged; 3 patients died of asphyxia due to long poisoning time. Two patients died of severe complications.

**Result:**

The total effective rate and oxygenation index of the study group were significantly different from those of the control group (*P* < 0.05).

**Conclusion:**

In the clinical nursing work of patients with severe carbon monoxide toxic pulmonary edema, the nursing effect of emergency cluster therapy is ideal. Patients with carbon monoxide poisoning have obvious age, gender, poisoning causes, and seasonal characteristics. It is an important means to carry out targeted publicity and education in daily life and take effective preventive measures to prevent carbon monoxide poisoning. Once poisoning occurs, timely treatment should be carried out, and careful nursing should be provided to help patients get rid of the danger.

## 1. Introduction

Gas poisoning is usually caused by carbon monoxide in the gas. Carbon monoxide (CO) is an odorless, nonirritating toxic gas with a molecular weight of 28.01. The main sources of CO are incomplete combustion of carbonaceous materials, vehicle exhaust, smoking, and so on. CO poisoning is easy to occur in car repair room or garage, toilet with gas water heater, and enclosed space with fireplace. Due to poor ventilation, if it is not found in time, it is easy to cause immediate death [1].

In clinic, severe carbon monoxide toxic pulmonary edema is prevalent, particularly in the winter. Acute hypoxia and enhanced pulmonary capillary permeability are the particular etiology, which is produced by inhaling a substantial quantity of carbon monoxide [2]. It produces noncardiogenic pulmonary edema in individuals and is a major danger to their health. Carbon monoxide poisoning has a protracted course and a sluggish recovery. Patients will develop delayed encephalopathy if therapy is not given promptly and thoroughly. As a result, it is critical to provide prompt treatment and attentive nursing to patients with carbon monoxide poisoning in order to enhance patient recovery and limit the risk of delayed encephalopathy. Pulmonary edema is a major symptom of lung damage in acute severe CO poisoning. Early onset, furious, and fast dissipation are all characteristics of pulmonary edema. The incidence rate is 10% ~30% [3]. In order to improve the quality of life of patients with acute carbon monoxide poisoning and make them recover as soon as possible, the author summarized the clinical data of 13 patients with acute carbon monoxide poisoning pulmonary edema in our hospital from January 2011 to April 2016 and exchanged treatment experience.

## 2. Materials and Methods

### 2.1. Research Objects

Methods from January 2011 to April 2016, 13 patients with acute CO toxic pulmonary edema were selected, including 8 males and 5 females, aged 32-76 years. The cause of poisoning in all patients was burning coal and charcoal in the family stove for heating. There was a clear history of CO exposure poisoning. It was estimated that the exposure time of CO was 8 ~ 32 h. There were 6 patients with severe poisoning, including coma, purplish or pale skin, and mucous membrane, weakening or even disappearing of various reflexes, incontinence of urine and urine, and increased muscular tension. The clinical manifestations of 31 patients with moderate poisoning were drowsiness, cherry red mucous membrane and nail bed, facial flushing, rapid pulse, tendon reflex, and pupil's slow light reflex. Headache, dizziness, exhaustion, vomiting, nausea, and other usual symptoms were experienced by 13 individuals with mild poisoning. During therapy, several patients were exposed to foam or pink foam sputum. There were a few cases of stomach contents or dark vomit. The breath on double lung auscultation was harsh, with a moist tone and/or wheeze, and the breathing rate rose 3246 times per minute. There was also sinus tachycardia, which ranged between 108 and 160 beats per minute. Six of the patients had cardiac failure, five had shock, and three had aspiration pneumonia. Type I respiratory failure was detected in 9 of the patients' arterial blood gases. On the basis of stable vital signs, all patients got a lung CT scan after admission. The lung texture was thickened and revealed ground glass-like alterations on a CT scan., especially in the upper lungs; the light transmittance of both lungs was decreased, and there were widely distributed nodular and patchy high density shadows and ground glass like shadows, with fuzzy edges, especially in the inner and middle zones of both lungs; accompanied by a small amount of pleural effusion (Figure 1).

### 2.2. First Aid and Nursing Methods

#### 2.2.1. First Aid

*(1) Evacuate the Patient from the Poisoning Site*. Immediately transfer the poisoned person to a place with air circulation. Make the patient lie flat, loosen the patient's trouser belt and clothing belt, remove the secretions in the mouth and nose, and keep the respiratory tract smooth. For patients with blurred consciousness, their heads should be tilted to one side to prevent asphyxia caused by aspiration of vomit.

*(2) Oxygen Supply*. In timely correction of patients with hypoxia, to prevent patients with brain cell lesions, the patients with mild and moderate poisoning should be put on nasal catheter or face mask and inhale 5-10 l/min high flow oxygen; for the patients with severe poisoning, the blood oxygen content and oxygen partial pressure should be increased, the hypoxia state of cells should be corrected, the dissociation of COHb should be promoted, and the occurrence of brain edema should be prevented.

*(3) Prevent Brain Edema*. For patients with severe coma or convulsion, ice bags can be placed on the head of patients to prevent brain edema.

#### 2.2.2. Nursing Methods

*(1) Hyperoxia Nursing*. The patients were given intravenous drip of 20% mannitol 250 ml or adenosine triphosphate, vitamin C, and cytochrome *c*. Once pulmonary edema was diagnosed, the foreign bodies in the oral cavity were removed immediately, and the oropharyngeal airway was unobstructed. In the early stage, the patients were given normal pressure mask, high flow oxygen inhalation, diuresis, dexamethasone, free radical scavenging, energy preparation, protection of gastric mucosa, maintenance of circulation, anti-infection, and other drugs. Treat the issue as soon as possible. Nine patients had endotracheal intubation and ventilator-assisted breathing, while four others received normal pressure mask high flow oxygen treatment. Five patients were treated with hyperbaric oxygen while their vital signs were somewhat stable. 48-hour hyperbaric oxygen treatment plan for 8 patients with unstable circulation: mild and severe poisoning patients received suitable hyperbaric oxygen therapy. When using high-capacity oxygen equipment, nursing personnel should inspect the device for defects, check for the presence of rescue medications and conduct a pressure test to alert patients to different potential discomforts. Nurses should tightly regulate the period of pressure and decompression before patients take hyperbaric oxygen, and the mask should be near to the patient's cheek to guarantee efficient oxygen inhalation. Sober patients were instructed to pinch their noses, close their mouths, blow, and swallow in the proper manner. The head should be tilted for patients who have lost consciousness. Hyperbaric oxygen treatment should be provided to patients with stable vital signs. The pressure of 0.20-0.25 MPa, pure oxygen should be inhaled for 30 min, twice, and the air in the cabin should be inhaled every 5 min, once a day, totally 1-2 times. When the patient increased the arterial oxygen partial pressure by 10 mmHg within 4 hours of treatment, it was judged to be effective. It is effective to increase the arterial partial pressure of oxygen by 10mmhg within 4H to 6 h. When the arterial oxygen partial pressure was increased by 10mmhg at 6 h, it was judged as invalid.

*(2) Mental Nursing*. Carbon monoxide poisoning patients will have a certain degree of self-care defects and physical discomfort, AND there will be fear, anxiety, pessimism, irritability and other negative emotions. Nurses should take appropriate psychological care of patients, take the initiative to care for patients, help patients, increase the number and time of ward visits, explain relevant disease knowledge to patients, introduce successful cases in the past, help them establish confidence in treatment, eliminate patients' fear and anxiety, and make them actively cooperate with the medical staff, shorten the time of recovery, and improve the prognosis.

*(3) Skin Care*. After a period of time, patients with carbon monoxide poisoning in the skin, heel blisters, and other impaired blood circulation. Doctors and nurses administer 0.5 percent iodophor to tiny blisters to aid absorption, disinfect big blisters as needed, and drain exudate with an aseptic syringe. Wipe the afflicted area with 0.5 percent iodophor after extraction. The diseased region may be treated twice a day with an infrared baking lamp and then covered with sterile gauze. To avoid aggravating skin injury, advise the patient to avoid dragging while rolling over.

*(4) Limb Function Recovery Nursing*. Nursing staff should assist patients to get out of bed early or massage patients properly, promote blood circulation of patients' limbs, control the time of each exercise of patients, and exercise their limbs fully and moderately to avoid fracture or dislocation.

(5) *Health Education for Patients*

Nursing staff should explain the harm of carbon monoxide poisoning to patients and inform patients that they should be treated in time after finding poisoning. The patients who use the stove in autumn and winter should be equipped with complete ventilation devices and corresponding protective equipment; for those who use gas, the gas pipes and equipment should be overhauled. At the same time, proper health education should be given to patients and their families.

#### 2.2.3. The Control Group Was Given Nursing Intervention

Patients were given routine nursing intervention, which included closely monitoring changes in patients' vital signs, emergency rescue nursing, blood gas analysis, and central venous pressure monitoring, according to the standardized process of hospital emergency rescue; patients in the study group were given routine nursing intervention + emergency cluster therapy, with the routine nursing intervention being the same as in the control group. Mix methylprednisolone, 6 percent hydroxyethyl starch sodium, 10% sodium chloride injection, and furosemide and then pump them at a rate of 200 ml/h. The daily dosages are 240 mg, 500 ml, 60 ml, and 100 mg, respectively..

### 2.3. Observation Index and Statistical Analysis

Respiratory rate, peripheral noninvasive oxygen saturation, arterial oxygen partial pressure/oxygenation index, carboxyhemoglobin, and other indicators were detected after 3 days of treatment; the clinical effect was observed; lung CT was reexamined after 3-5 days of treatment. One dead patient was not given index statistics. Statistical analysis: SPSS13.0 software was used for statistical analysis. Measurement data mean standard deviation ($\bar{x}\pm s$) expressed by *t*-test, *P* < 0.05, for the difference was statistically significant.

## 3. Result

Changes of respiratory rate, arterial oxygen partial pressure ,and carboxyhemoglobin: the respiratory indexes of 12 patients were gradually stable 48 hours after comprehensive treatment, and the peripheral noninvasive oxygen saturation was in the normal range. After treatment, respiratory rate and carboxyhemoglobin were significantly decreased, arterial oxygen partial pressure was significantly increased, the differences were statistically significant (*P* < 0.05), as Table 1 shows.

### 3.1. CT Findings of Lung

Pulmonary CT scan was reexamined 3-5 days after poisoning, and the high density of pulmonary edema disappeared in 10 patients (Figure 1(b)). Two patients left high-density consolidation shadow in both lungs, especially in the right upper lung (Figure 2(b)). After strengthening anti-infection, atomization, and physical vibration, the course of disease was 10-14 days, and CT scan showed that the high-density patchy shadow was alleviated or disappeared.

### 3.2. Clinical Effect

Seven of the nine patients with endotracheal intubation and ventilator-assisted breathing were taken offline to resume self-help breathing within 24 hours, with five of them extubated within 24 hours, two extubated within 48 hours, one taken off-line to resume spontaneous breathing within 48 hours, and one dying of severe heart failure within 48 hours.

### 3.3. Control Results

Compared with the control group, the total effective rate and oxygenation index of the study group were significantly different (*P* < 0.05), with statistical significance. Refer to Table 2 for details.

## 4. Conclusion

There are many mechanisms of pulmonary edema induced by acute carbon monoxide poisoning, the most important of which are hypoxia and neurogenic edema. When CO is poisoned, the permeability of pulmonary capillaries is enhanced due to acute hypoxia and direct cytotoxic effect of CO, resulting in excessive overflow of intravascular fluid and destroying the dynamic balance of intravascular and extravascular fluid. When the amount of overflow exceeds the reflux capacity of lymphatic system, the edema fluid can gather in the pulmonary interstitium and alveoli, resulting in pulmonary edema. At the same time, CO poisoning causes a sudden increase in intracranial pressure, resulting in hypothalamic dysfunction; the body's stress response activates the sympathetic nerve; the release of a large number of adrenergic neurotransmitters causes strong contraction of peripheral blood vessels, resulting in a large number of blood transfers from high resistance systemic circulation to low resistance pulmonary circulation, and the patients' pulmonary capillary permeability increases; the patients' pulmonary capillary appropriate treatment strategies should be chosen based on the real condition of individual patients in order to get the optimal therapeutic impact. When the patient's condition allows, hyperbaric oxygen should be used initially. The pressure in the airway and alveoli rises when patients are given hyperbaric oxygen, and the pressure between the lung tissues rises as well. When the hydrostatic pressure between the lung tissues surpasses the hydrostatic pressure in the capillaries, liquid extravasation in the capillaries is prevented, lymphatic reflux is enhanced, and edema between the tissues is promptly controlled. At the same time, hyperbaric oxygen therapy can improve the hypoxia state of various organs and tissues, enhance aerobic oxidation of tissues and cells, weaken anaerobic digestion, increase energy, reduce acid metabolites, restore ion disorder inside and outside cells, and reduce edema inside and outside cells.

In the treatment of hyperbaric oxygen in acute stage of CO poisoning, the author selected 0.20-0.25 MPa pressure treatment for 1-2 times, which can reduce the degree of pulmonary edema while completely excluding CO in vivo. As the results show, the wet sound of the double lung disappeared from the third to fifth day after poisoning. The high-density imaging manifestations of pulmonary edema disappeared after reexamination of lung CT. When the patients with severe pulmonary edema after acute CO poisoning are treated with hyperbaric oxygen, special attention should be paid to the occurrence of pulmonary edema rebound after decompression. This situation is reported very little at home and abroad, but in the actual clinical work [4–6]. The patients had a shortness of breath during decompression, and the respiratory emergency continued to worsen after leaving the cabin. The respiratory distress needed to consider the pulmonary edema and rebound. The main mechanism may be that the lung tissue, capillary endothelial cells, pulmonary epithelial cells, and so on have not been completely repaired [7–9]. During decompression, the vessels are diastolic and permeability increase, while the pressure in the airway decreases, the static pressure in the capillary is relatively high, the fluid in the vessels is easy to exude, which leads to the pulmonary edema more severe than the pressure and pressure stabilization, and reduces the decompression speed; after leaving the cabin, according to the patient, the pressure is increased according to the patient The patients were treated with symptoms, such as sitting position, high flow oxygen inhalation, and diuresis, and tracheal intubation and ventilator assisted breathing if necessary. For the patients with severe CO poisoning, it is not suitable for hyperbaric oxygen treatment, and there are respiratory distress and unstable vital signs. According to the treatment principle of acute respiratory distress syndrome, we can conduct protective ventilation intermittent pure oxygen therapy [10–12].

In this group of cases, 8 patients were not suitable for emergency hyperbaric oxygen treatment, they were given endotracheal intubation, ventilator assisted breathing, positive end expiratory pressure + low tidal volume ventilation, according to the patient's symptoms, signs, and blood gas analysis results, early ventilator treatment, and early extubation principle, or they were given normal pressure mask oxygen. Similarly, after treatment, the respiratory rate of the patient decreased significantly, and the carboxyhemoglobin basically returned to normal; on the third to fifth day after poisoning, the signs of pulmonary edema basically disappeared, and the signs of pulmonary edema basically disappeared after reexamination of lung CT, reaching the expected therapeutic effect: glucocorticoid in the treatment of brain edema, but also can reduce the degree of pulmonary edema, mainly antagonize the body's systemic inflammatory response, inhibit the release of inflammatory factors, reduce the production of platelet activating factor and oxygen free radicals, protect cell membrane, improve capillary permeability, and reduce fluid leakage [13–15].

Furthermore, glucocorticoids may aid in the absorption of lung interstitial fluid, the secretion of surfactant by alveolar type II cells, the relief of bronchospasm, the inhibition of pulmonary fibrosis, and other activities. The author selected dexamethasone 5-15 mg for therapy because it has a higher anti-inflammatory impact and can better control systemic inflammatory response than hydrocortisone and methylprednisolone. At the same time, the preservation of the stomach mucosa should be prioritized. Aspiration pneumonia refers to the inhalation of foreign bodies into the trachea, bronchus, and lung, causing bronchiole obstruction and distal lung tissue collapse; with the foreign body into the bacteria in the lung symptoms, lung signs, whether to inhale food residues during endotracheal intubation, lung CT imaging performance, can basically judge whether there is aspiration pneumonia. However, in the absence of medical history, intratracheal food residue, and other factors, CT imaging alone may be difficult to distinguish.

For patients with inhalation pneumonia caused by CO poisoning, the first thing is to keep the respiratory tract unobstructed, endotracheal intubation should be given according to the condition, and ventilator-assisted breathing should be given when necessary. Secondly, studies have shown that the pathogen of aspiration pneumonia is often mixed infection [16]. Therefore, when selecting antibiotics, we need to choose broad-spectrum antibiotics, which can cover positive cocci, negative bacilli, especially anaerobic bacteria, such as carbapenems, or choose antibiotics according to the results of pathogen culture. In addition, comprehensive application of hormone, bronchoscopic sputum suction, bronchoalveolar lavage, ammonia brominated sputum, systemic nutritional support, turning over and slapping back, airway nursing, and other treatments is needed to promote the improvement and healing of aspiration pneumonia. After treatment, 3 cases still had high-density patchy shadow. Combined with the history of vomiting, it was confirmed that they were complicated with aspiration pneumonia.

Severe carbon monoxide poisoning is a common toxic disease in clinic, which can cause hypoxic injury of multiple systems and organs in the whole body, cause pulmonary edema, and seriously threaten the life safety of patients. According to relevant literature research and reports, the pathogenesis of severe carbon monoxide toxic pulmonary edema is as follows: first, hypoxia, when poisoning occurs, the patient inhales a large amount of carbon monoxide, causing it to quickly diffuse into the blood through the patient's lung [17], organically combine with hemoglobin in the blood, so that hemoglobin loses its oxygen carrying capacity. The produced carboxyhemoglobin not only has no oxygen carrying capacity but also affects the dissociation of oxyhemoglobin, which leads to cell dysfunction and makes the body in a state of severe hypoxia and energy metabolism disorder [18, 19], resulting in pathological injury. Furthermore, when a patient is in a toxic state, the permeability of the lung capillary wall and alveolar wall is increased, the vascular endothelium swells, the lymphatic circulation is blocked, and edematous fluid collects in the patient's lung interstitium and alveoli, causing asphyxia and coma; second, inflammatory reaction, after poisoning, the patient will activate inflammatory cells, which can promote the release of inflammatory. The organic combination of oxidases causes electron transmission to be obstructed and oxidative phosphorylation to be blocked in the respiratory chain, resulting in energy metabolism disturbance and pathological damage; fourth, carbon monoxide may disrupt mitochondrial function by binding heme protein. A large number of clinical studies have confirmed that emergency cluster therapy for patients with severe carbon monoxide toxic pulmonary edema can significantly improve the clinical symptoms of wheezing, chest tightness, and dyspnea, shorten the course of disease, and improve the prognosis of patients.

In this study, the total effective rate and oxygenation index of the study group were 100.00% and (203.5 ± 19.2), respectively, which were significantly better than those of the control group. Based on the above theory, the application of emergency cluster therapy in the clinical nursing of patients with severe carbon monoxide toxic pulmonary edema has ideal nursing effect and can significantly improve the oxygenation index of patients, which is worthy of clinical reference and promotion.

## Figures and Tables

**Figure 1:** CT image of pulmonary edema caused by carbon monoxide poisoning.

**Figure 2:** CT image of lung in patients with carbon monoxide poisoning and aspiration pneumonia.

**Table 1:** Changes of respiratory rate, arterial oxygen partial pressure, and carboxyhemoglobin before and after treatment ($\bar{x}\pm s$, *n* = 12 in each group).

Index	Before therapy	After treatment
Respiratory rate (times/min)	35.92 ± 4.27	30.67 ± 2.53
Arterial partial pressure of oxygen (mmhg)	55.5 ± 5.66	84.08 ± 14.47
Carboxyhemoglobin (%)	39.75 ± 11.29	2.58 ± 1.56

**Table 2:** Comparison of nursing effect between the two groups.

Group	Number of cases	Remarkable effect	Effective	Invalid	Total effective rate of nursing	Oxygenation index
Research group	19	12	7	0	100%	203.5 ± 19.2
Control group	19	6	8	5	73.68%	260.2 ± 22.2
$\frac{x^{2}}{t}$					5.7576	8.4204
*P*					< 0.05	< 0.05

## Data Availability

The data used to support the findings of this study are included within the article.
